The article "Colonic Gallstone Ileus: A Rare Etiology of Large Bowel Obstruction" was retracted in 2024. Reasons: false authorship; unreliable results or conclusions; no approval from an author; concerns about the authorship.

# Colonic Gallstone Ileus: A Rare Etiology of Large Bowel Obstruction

**DOI:** 10.7759/cureus.20338

**Published:** 2021-12-10

**Authors:** Abdulaziz O Alshehri, Turki S Aljuhani, Salihah S Alotaibi, Shahad A Almughamisi, Mariam M Ageel, Abdulmuhsen H Alameer, Khalid M Alqahtani, Ziyad A Alhumaid, Abdullah S Alsuwayeh, Mohammmad S Almarri, Saja F Almotadaris, Hamad Y Alsaeed, Abdallh M Alatwai, Ahmed M Alatawi, Faisal Al-Hawaj

**Affiliations:** 1 College of Medicine, University of Debrecen, Debrecen, HUN; 2 College of Medicine, University of Hail, Hail, SAU; 3 College of Medicine, AlMaarefa University, Ad Diriyah, SAU; 4 College of Medicine, King Abdulaziz University, Jeddah, SAU; 5 General Practice, Al-Ahsa Health Cluster, Al-Ahsa, SAU; 6 College of Medicine, King Khalid University, Abha, SAU; 7 College of Medicine, King Saud bin Abdulaziz University for Health Sciences, Riyadh, SAU; 8 College of Medicine, Imam Mohammed Ibn Saud Islamic University, Riyadh, SAU; 9 General Surgery, Adan Hospital, Hadiya, KWT; 10 Unaizah College of Medicine, Qassim University, Qassim, SAU; 11 College of Medicine, Jordan University of Science and Technology, Irbid, SAU; 12 College of Medicine, Tabuk University, Tabuk, SAU; 13 College of Medicine, Imam Abdulrahman Bin Faisal University, Dammam, SAU

**Keywords:** case report, gallbladder disease, gallstone, large bowel obstruction, cholecystocolic fistula

## Abstract

Large bowel obstruction is a surgical emergency that requires prompt diagnosis and management. It is frequently caused by colon cancer. However, the common benign etiologies include volvulus, hernia, adhesions, and strictures. Imaging studies are essential to establish the diagnosis and identify the etiology. We present the case of a 44-year-old female who presented to the emergency department with abdominal pain and distension for a one-week duration. The pain was associated with decreased bowel motions and vomiting. Her past medical history was significant for diabetes mellitus, dyslipidemia, polycystic ovarian syndrome, and recurrent episodes of biliary colic. Upon examination, she had tachycardia, normal temperature, and normal blood pressure. Abdominal examination revealed a distended abdomen with generalized tenderness and increased intensity of bowel sounds. The laboratory markers were noncontributory. Abdominal computed tomography (CT) scan of the abdomen with intravenous contrast demonstrated the presence of an oval-shaped hypodense intraluminal mass in the sigmoid colon where there was a transition point with proximal colonic dilatation. There was an abnormal communication between the gallbladder and the colon at the hepatic flexure, representing a cholecystocolic fistula tract. This represents a mechanical obstruction of the large bowel due to migrated gallstone through a cholecystocolic fistula tract. The patient was prepared for an emergency laparotomy. The gallstone was removed, and the sigmoid colon was sutured primarily. Resection of the gallbladder was made with the closure of the fistula tract. Following the surgery, the patient reported a resolution of her abdominal pain. Oral feeding was started gradually. After six months of close follow-up, the patient remained asymptomatic with no new complaints. Cholecystocolic fistula is a very rare complication of gallbladder disease. Despite its rarity, surgeons should remember this etiology of large intestinal obstruction when they encounter a patient with gallbladder disease.

The article "Colonic Gallstone Ileus: A Rare Etiology of Large Bowel Obstruction" was retracted in 2024. Reasons: false authorship; unreliable results or conclusions; no approval from an author; concerns about the authorship.

## Introduction

Large intestinal obstruction accounts for one-fourth of all bowel obstructions. The most common etiology of large bowel obstruction is malignancy [1]. The benign causes include volvulus, hernia, adhesion, and stricture. The diagnosis of large bowel obstruction can be suspected based on the clinical presentation, but imaging studies are key to confirming the diagnosis. A computed tomography (CT) scan is the modality of choice as it can confirm the diagnosis, localize the obstruction, and identify the etiology. Here, we present the case of a middle-aged woman with a history of gallbladder disease who developed large intestinal obstruction secondary to obstructive gallstone from cholecystocolic fistula. This unique etiology of large bowel obstruction is very rare and poses a diagnostic challenge. While gallbladder stones are very common and affect up to 10% of women [2], cholecystocolic fistula is considered a very rare complication of gallbladder disease.

## Case presentation

We present the case of a 44-year-old female who presented to the emergency department complaining of abdominal pain for the last six days. The pain was generalized and had colicky nature. She had the pain every three to four hours and partially resolved after taking over-the-counter antispasmodic agents. The pain was radiating to the right shoulder. The pain was moderate in severity, and she scored it as 6 on the 10-point severity scale. She reported that the pain gets worse after food intake. The patient also complained of abdominal distension, nausea, vomiting, and decreased bowel motions. She had not passed stools or even gases for the last two days. The patient did not report any history of weight loss or decreased appetite.

The past medical history was remarkable for diabetes mellitus, dyslipidemia, and secondary infertility secondary to polycystic ovarian syndrome. The patient was morbidly obese with a body mass index of 41 kg/m^2^. She had multiple episodes of biliary colic due to gallstone. She was planned to have an elective laparoscopic cholecystectomy, but the patient refused the surgery at this time due to fear of encountering coronavirus disease 2019 (COVID-19) during hospitalization. Her medications include atorvastatin 20 mg, glipizide 2.5 mg, metformin 500 mg, perindopril 5 mg, and aspirin 75 mg. She was not known to have any food or drug allergies. She worked as a school teacher. She never smoked or consumed alcohol. The family history was remarkable for glucose-6-phosphate dehydrogenase deficiency.

The article "Colonic Gallstone Ileus: A Rare Etiology of Large Bowel Obstruction" was retracted in 2024. Reasons: false authorship; unreliable results or conclusions; no approval from an author; concerns about the authorship.

Upon examination, the patient appeared in pain. She was not having any signs of respiratory distress. The vital signs indicated tachycardia (110 bpm), normal respiratory rate (15 bpm), elevated blood pressure (140/85 mmHg), and normal temperature (37.1°C). Abdominal examination revealed a distended abdomen with generalized tenderness. No guarding or rigidity was appreciated. Bowel sounds were of increased intensity and frequency. Digital rectal examination revealed an empty rectum. Examination of other systems yielded normal findings.

Initial laboratory investigation, including hematological and biochemical parameters, did not reveal any abnormalities. It revealed a hemoglobin level of 13.9 g/dL, leukocyte count of 8400/μL, and platelet count of 380,000/μL. Renal function tests, including blood urea nitrogen (10 mg/dL) and creatinine (0.8 mg/dL), were within the normal limits. Liver enzymes were not elevated (Table 1).

**Table 1:** Summary of the results of the laboratory findings

Laboratory Investigation	Unit	Result	Reference Range
Hemoglobin	g/dL	13.9	13–18
White Blood Cell	1000/mL	8.4	4–11
Platelet	1000/mL	380	140–450
Erythrocyte Sedimentation Rate	mm/hour	12	0–20
C-Reactive Protein	mg/dL	8.1	0.3–10
Total Bilirubin	mg/dL	1.1	0.2–1.2
Albumin	g/dL	3.8	3.4–5
Alkaline Phosphatase	U/L	51	46–116
Gamma-glutamyltransferase	U/L	23	15–85
Alanine Transferase	U/L	20	14–63
Aspartate Transferase	U/L	17	15–37
Blood Urea Nitrogen	mg/dL	10	7–18
Creatinine	mg/dL	0.8	0.7–1.3
Sodium	mEq/L	138	136–145
Potassium	mEq/L	3.9	3.5–5.1
Chloride	mEq/L	105	98–107

The patient underwent a computed tomography scan of the abdomen with intravenous contrast. The scan demonstrated the presence of an oval-shaped hypodense intraluminal mass in the sigmoid colon where there was a transition point with proximal colonic dilatation. There was an abnormal communication between the gallbladder and the colon at the hepatic flexure, representing a cholecystocolic fistula tract. Multiple outpouchings from the colon were noted in the sigmoid colon in keeping with uncomplicated diverticulosis. The aforementioned findings represent a mechanical obstruction of the large bowel due to migrated gallstone through a cholecystocolic fistula tract (Figures 1-2). 

The article "Colonic Gallstone Ileus: A Rare Etiology of Large Bowel Obstruction" was retracted in 2024. Reasons: false authorship; unreliable results or conclusions; no approval from an author; concerns about the authorship.

**Figure 1:** Coronal CT image demonstrates the gallstone (arrow) within the lumen of the sigmoid colon CT: computed tomography

**Figure 2:** Sagittal CT image demonstrates the fistula tract (arrow) between the gallbladder and the colon CT: computed tomography

The patient was prepared for an emergency laparotomy. The operation was conducted under general anesthesia, and the patient was in the supine position. During exploration, the point of transition was identified. The gallstone was removed, and the sigmoid colon was sutured primarily (Figure 3). Resection of the gallbladder was made with the closure of the fistula tract. The operation lasted for three hours, and the estimated blood loss was 50 mL. The patient had an uneventful recovery.

**Figure 3:** Gross pathology image of the removed gallstone

Following the surgery, the patient reported a resolution of her abdominal pain. Oral feeding was started gradually. The patient was tolerating the feeding with no complaints. She was discharged on the fifth postoperative day after eight days of hospitalization. After six months of close follow-up, the patient remained asymptomatic with no new complaints.

## Discussion

We presented the case of a cholecystocolic fistula resulting in large intestinal obstruction due to a migrated gallstone. Cholecystocolic fistula is among the rare and late complications of gallbladder disease. It accounts for less than 20% of all cholecystoenteric fistulas. Previous research suggested that it is encountered in one per 1,000 of cholecystectomy operations [3]. In our case, the patient's age was relatively younger than what is commonly reported. Previous data on this condition typically presents in the elderly population with a mean age of 70 years [4].

Certain conditions were found to increase the risk of the formation of cholecystoenteric fistulas. Such factors include previous gastric surgery, abdominal trauma, duodenal ulcer, and cholecystostomy. In our patient, however, she did not have any history of these conditions, and the fistula formed spontaneously. Regarding the clinical manifestation, diarrhea was reported as the most frequent symptom. Abdominal pain, fever, and jaundice have been reported. However, less than 20% of patients present with large bowel obstruction, as in our case.

It is interesting to note that less than 10% of patients with cholecystocolic fistula had been diagnosed preoperatively [4]. The diagnosis is often made during the operation. Ultrasound has a limited role in establishing this diagnosis. In some cases, the diagnosis was established by barium enema [5]. In the present case, the diagnosis was made accurately by the computed tomography scan of the abdomen, and the fistula tract was well appreciated.

The article "Colonic Gallstone Ileus: A Rare Etiology of Large Bowel Obstruction" was retracted in 2024. Reasons: false authorship; unreliable results or conclusions; no approval from an author; concerns about the authorship.

The standard treatment of cholecystocolic fistula includes cholecystectomy and closure of the fistula tract. The surgery is performed laparoscopically [5]. However, laparoscopic procedures for such conditions have been associated with a high conversion rate to open laparotomy and prolonged operative time [4].

## Conclusions

Cholecystocolic fistula is a very rare complication of gallbladder disease. Despite its rarity, surgeons should remember this etiology of large intestinal obstruction when they encounter a patient with gallbladder disease. The diagnosis may be made preoperatively with a computed tomography scan, which can demonstrate the fistula tract. Cholecystectomy and closure of the fistula is the management of choice.

## References

[1] Kahi CJ, Rex DK (2003). Bowel obstruction and pseudo-obstruction. Gastroenterol Clin North Am.

[2] Zeng Q, He Y, Qiang DC, Wu LX (2012). Prevalence and epidemiological pattern of gallstones in urban residents in China. Eur J Gastroenterol Hepatol.

[3] Agrawal V, Joshi U, Manandhar S (2017). Spontaneous cholecystocolic fistula: an uncommon complication of chronic cholecystitis. Clin Case Rep.

[4] Costi R, Randone B, Violi V (2009). Cholecystocolonic fistula: facts and myths. A review of the 231 published cases. J Hepatobiliary Pancreat Surg.

[5] Gibreel W, Greiten LL, Alsayed A, Schiller HJ (2018). Management dilemma of cholecysto-colonic fistula: case report. Int J Surg Case Rep.

